# The Arctic charr (*Salvelinus alpinus*) genome and transcriptome assembly

**DOI:** 10.1371/journal.pone.0204076

**Published:** 2018-09-13

**Authors:** Kris A. Christensen, Eric B. Rondeau, David R. Minkley, Jong S. Leong, Cameron M. Nugent, Roy G. Danzmann, Moira M. Ferguson, Agnieszka Stadnik, Robert H. Devlin, Robin Muzzerall, Michael Edwards, William S. Davidson, Ben F. Koop

**Affiliations:** 1 Fisheries and Oceans Canada, Centre for Aquaculture and Environmental Research, West Vancouver, British Columbia, Canada; 2 University of Victoria, Department of Biology, Victoria, British Columbia, Canada; 3 Simon Fraser University, Molecular Biology and Biochemistry, Burnaby, British Columbia, Canada; 4 University of Guelph, Department of Integrative Biology, Guelph, Ontario, Canada; 5 Icy Waters Ltd, Whitehorse, Yukon, Canada; University of Iceland, ICELAND

## Abstract

Arctic charr have a circumpolar distribution, persevere under extreme environmental conditions, and reach ages unknown to most other salmonids. The *Salvelinus* genus is primarily composed of species with genomes that are structured more like the ancestral salmonid genome than most *Oncorhynchus* and *Salmo* species of sister genera. It is thought that this aspect of the genome may be important for local adaptation (due to increased recombination) and anadromy (the migration of fish from saltwater to freshwater). In this study, we describe the generation of a new genetic map, the sequencing and assembly of the Arctic charr genome (GenBank accession: GCF_002910315.2) using the newly created genetic map and a previous genetic map, and present several analyses of the Arctic charr genes and genome assembly. The newly generated genetic map consists of 8,574 unique genetic markers and is similar to previous genetic maps with the exception of three major structural differences. The N50, identified BUSCOs, repetitive DNA content, and total size of the Arctic charr assembled genome are all comparable to other assembled salmonid genomes. An analysis to identify orthologous genes revealed that a large number of orthologs could be identified between salmonids and many appear to have highly conserved gene expression profiles between species. Comparing orthologous gene expression profiles may give us a better insight into which genes are more likely to influence species specific phenotypes.

## Introduction

In frigid conditions, too cold for other freshwater fish species, Arctic charr can survive and flourish [1,2]. Arctic charr hold the record for the most northern freshwater fish, with populations found in lakes on the northern reaches of Ellesmere Island in the Canadian territory of Nunavut [3–5]. Increased survival of Arctic charr in cold seawater relative to other salmonids (Atlantic salmon, brook, brown, and rainbow trout) is likely due to increased plasma electrolyte levels and characteristics of their epidermal layer that prevents plasma ice crystallization [6].

Arctic charr possess remarkable physiological, morphological, behavioural and life-history variation throughout their circumpolar distribution. Arctic charr from different populations, and even those within the same lake, are phenotypically diverse—an observation which has prompted the suggestion that they are the most variable vertebrate species [7]. Freshwater populations often contain resource-based morphs that vary in the degree of morphological, life-history, and genetic differentiation. Diversity between and among populations has led to challenges in determining taxonomic designations within the species complex, which has complicated legislative approaches to the conservation of this charismatic species [8].

Arctic charr have been an important food resource for people in the Canadian Arctic for thousands of years. More recently, the species has been cultured in commercial operations at more southern latitudes, but the industry is relatively undeveloped compared to that of other salmonids such as Atlantic salmon or rainbow trout. Arctic charr culture in Canada is based on three commercial strains (Nauyuk Lake and Tree River strains from Nunavut, and the Fraser River strain from Labrador). The strains were established from wild collections in the late 1970’s and early 1980’s, and are genetically differentiated from one another due to their different evolutionary and cultural legacies [9]. The Nauyuk and Tree River populations belong to the Arctic phylogeographic group, whereas the Fraser strain is from the Atlantic group [10,11].

Akin to other salmonids, Arctic charr have extensive duplicated regions of their genomes stemming from a salmonid-specific genome duplication that occurred ~90 million years ago in the common ancestor to the salmonids [12,13]. Recombinations between homeologous chromosomes (i.e. chromosomes duplicated during the genome duplication) have lead to relatively high sequence similarity and complex segregation patterns between chromosomes, which in turn complicates the construction of genetic linkage maps [14–19], genetic analyses [16], and assembling the genome. In addition to the duplicated nature of their genome, salmonids also show evidence of chromosomal rearrangements that arose after the duplication event.

Two main karyotypes are present in salmonids (though there are others), based on the number of fusions found between chromosomes [20,21]. The “A” karyotype is commonly comprised of 80 chromosomes with a total of 100 chromosome arms (*Salvelinus*), and the “B” karyotype is customarily formed from 60 chromosomes and 104 chromosome arms (*Oncorhynchus* and *Salmo*) [21]. The Arctic charr retain the “A” karyotype with 78 chromosomes (n = 39) and 98 chromosome arms [20]. Based on these observations, researchers have inferred that Robertsonian-like translocations/fusions are less common in *Salvelinus* compared to *Oncorhynchus* [14,20], which suggests that *Salvelinus* has a less derived (more basal) genomic structure.

The number of chromosomes or chromosome arms may influence the rate of recombination between non-sister chromatids and consequently the rate of fixation for new mutations. With additional chromosomes, chromosome arms, and fewer Robertsonian translocations, the “A” karyotype might be expected to have higher levels of chiasmata formation and additional recombination events [20,22,23]. Based on this hypothesis, this would potentially result in greater nucleotide variation that is fundamental to adaptation to many different locations [20,22]. Conversely, a greater recombination frequency would lower levels of linkage disequilibrium that underlies local adaptation [20,22]. Robertsonian translocations may also alter the nuclear architecture of “B” karyotypes [24].

In the present study, we built a new genetic linkage map derived predominantly from the Nauyuk and Tree River strains. We sequenced several genomic libraries, with both short and long read technologies, and assembled these into an initial whole genome assembly. The assembled genomic sequences were arranged into chromosomes using a previous genetic map (Fraser River strain [15]), our new genetic map, and support from synteny with the rainbow trout genome assembly. With the resulting reference genome assembly, we performed several analyses in order to assess the completeness of the genome assembly, identify duplicated regions, and characterize repetitive DNA elements in the Arctic charr genome. RNA-seq was performed on 12 Arctic charr tissues to facilitate gene identification and to measure gene expression. We identified orthologous chromosomes in Arctic charr, northern pike [25], Atlantic salmon [26], coho salmon (unpublished GenBank version), rainbow trout (unpublished GenBank version), and Chinook salmon [27]. Orthologous genes (and homeologous genes within the Arctic charr genome) were then identified between these species based on the location of the genes between orthologous chromosomes (synteny) and protein similarity. Gene expression from multiple tissues was compared between orthologs and homeologs to first characterize the overall correlation between them, and then to identify genes that have expression profiles unique to Arctic charr as these genes have a greater chance of influencing traits specific to Arctic charr. In a final analysis, nucleotide variation was assessed in two commercial strains (Tree River and Nauyuk Lake) to determine how much variation might exist between these strains.

## Materials and methods

### Genetic map

#### Samples and library preparation

Fin clips and gender information was collected from eleven families of Arctic charr (Table 1). The families were generated from backcrosses of Nauyuk Lake and Tree River Arctic charr in 2001 [28], and were reared at Icy Waters Limited (Whitehorse, Canada [29]). In addition, two families were generated from Fraser river strains [30]. Seven of the families had a genetic background of Nauyuk Lake (female) x Tree River (male) hybrid females crossed to Tree River males. Two of the families had the same female maternal background, but were crossed to Nauyuk Lake males. Finally, two families were generated from crosses between Fraser River and Nauyuk Lake used in [30]. Animals were reared and sampled in compliance with the Simon Fraser University animal care protocol #1155MB-08. Fish were anesthetized with MS-222, or when euthanasia was necessary, fish were over-anesthetized with MS-222.

**Table 1:** Arctic charr genetic map crosses.

Family	1	2	3	4	5	7	9	52	59	F2	F3
Female	Hybrid NL_f_ x TR_m_									FR_u_ x NL_u_	FR_f_
Male	TR_m_							NL_m_		FR_m_	FR_u_ x NL_u_
Progeny	14	23	28	31	24	24	25	33	36	29	38

NL, Nauyuk Lake; TR, Tree River; FR, Fraser River (Labrador); m:male f:female u:unknown

A Gentra Puregene Tissue Kit (Qiagen, Venlo, Netherlands) was used to isolate DNA from ethanol-preserved fin clips. Some DNA samples were already extracted from previous studies [28,30]. DNA quality was verified on a 2% agarose gel and samples with poor quality DNA were not used. DNA concentration was normalized among samples that were going to be multiplexed.

For each sample, a modified two restriction enzyme RAD-sequencing protocol [31] was used to create an Illumina sequencing library (see [32] for details). Briefly, each DNA sample was added to a restriction-ligation mixture containing MseI and SbfI restriction enzymes as well as corresponding adapters with overhanging MseI or SbfI complementary sequence. The SbfI adapter contained a barcode for identifying sequences from that sample after multiplexing. A small amount of this mixture was then PCR amplified (16 cycles) using primers with sequence complementary to adapter sequences and overhangs with sequence necessary for Illumina sequencing. The quality of the amplification products were individually verified using agarose gel electrophoresis (1% gel). Multiple amplifications of a sample were added together for poorly amplifying samples.

The individual samples were then pooled into four different libraries (individuals per pool ranged from 74–87) and the volume of each pool was reduced using a SpeedVac (Labconco, Kansas City, MO). Agarose gel electrophoresis (1%) was used to exise a section of DNA from the pooled samples of approximately 450–700 nucleotides. This section was purified using a NucleoSpin Gel and PCR Clean-up kit (Macherey-Nagel, Bethlehem, PA). The size and quality of each library was assessed on a Fragment Analyzer (Advanced Analytical Technologies, Inc. Ankeny, USA). Four multiplexed libraries were created in this manner, and each library was sequenced at UC Berkeley's Vincent J. Coates Genomics Sequencing Laboratory on a HiSeq2500 using the rapid-run mode PE 150.

#### Data processing and genetic map construction

Reads were demultiplexed and quality control was performed using the process_radtags command in Stacks version 1.46 [33]. The following options were used: -q, -r, and -e sbfI. For all individuals, the ustacks command was then used to identify stacks with the following parameters: -m 3, -M 3, -N 3—max_locus_stacks 2 -H, and -p 4. A catalog was created using all of the parents (samples for the FamF2 and FamF3 dames were unavailable) with the cstacks command in combination with the -n 2 and -p 4 options. All individuals were then genotyped using the populations command and the—vcf, -t 4, and -m 6 parameters. The marker sequences were also exported with the—ordered_export and—fasta options for the populations command.

In order to address the missing FamF2 and FamF3 dames, a custom script was used to add a missing value for these individuals at each polymorphic genomic locus in the combined vcf file generated by Stacks (S1 File) (these were not used by the mapping software and only served as blank spaces). A file was also manually created with family information, to be used by the LepMap3 [34] software. The vcf file and family information were used to call missing parent genotypes with the ParentCall2 module of LepMap3 using the vcfFile option (all families together). Markers were then filtered based on segregation distortion (deviations from Mendelian inheritance) using a dataTolerance of 0.001 with the Filtering2 module.

LOD values from 8–40 (with a step of 1) were used to separate the markers into linkage groups with the SeparateChromosomes2 module and using the sizeLimit option set to 15 (similar to [14]). A sizeLimit of 15 removed most of the small linkage groups while retaining the largest and expected 39 linkage groups. Next, the genetic markers on the different LOD separated maps were ordered using the OrderMarkers2 module (male and female map combined). The ordered genetic markers (sequences were extracted using custom scripts) were aligned to the rainbow trout genome assembly (NCBI accession: GCA_002163495.1) using default setting of bwa mem [35]. These alignments were filtered (min mapq score of 30) and formatted using a custom script to only return a best alignment, and they were then visualized in R [36] using ggplot2 [37].

LOD scores for specific linkage groups were chosen to optimize the number of groups while minimizing the unnecessary removal of markers (based on the alignment of a linkage group to a rainbow trout chromosome—similar to [14]). Linkage groups were combined into a framework genetic map, and the JoinSingles2All module was used to add additional markers to this framework with a lodLimit of 10 and a lodDifference of 5. Each linkage group was then ordered six times with OrderMarkers2, and the best order (marker linearity in comparison to the rainbow trout genome assembly) was chosen as the final order. A comparison was performed between the updated genetic map from [15], and the current genetic map. This comparison shows the alignments of the genetic markers from both genetic maps to the Arctic charr genome assembly (described below). The chromosomal names were taken from the [15] genetic map.

To locate the sex determining region of the genome, a genome wide association test was performed with gender as the trait of interest (n = 232, families 52 and 59 did not have this metadata available). The vcf file, output from stacks, was modified to include linkage group information and marker order information with a custom python script (S1 File). The parents were removed from the vcf file with vcftools [38]. Plink v1.90b4.4 [39,40] was used to perform the association test with the following options:—allow-extra-chr,—allow-no-sex,—assoc, and—chr-set 39 no-xy. A Bonferroni correction was used to determine significance (0.05 alpha level/ 4677 variants = 0.000010691, or -log10(p) = 4.97).

### Genome assembly

#### Samples and library preparation

A single Arctic charr individual (female—inferred from the absence of the male-specific SDY gene in the sequence data set) of approximately 20 cm in length was obtained from Icy Waters Ltd. Tissues (eye, heart, spleen, gut, muscle, brain, hind kidney, head kidney, stomach, gill, liver, and gonad) were dissected from the female and stored in RNAlater (at -80°C) for RNA-seq analysis (see the *RNA-seq and gene annotation* section for RNA-seq information). The remaining tissues were also stored in RNAlater, and liver from this remaining tissue was used as the primary source for the DNA extraction. The DNA extraction followed the phenol extraction with Shepherd's crook method of Sambrook and Russell [41]. All animals were reared and sampled in compliance with the Simon Fraser University animal care protocol #1155MB-08.

Illumina library preparations and sequencing were performed by the McGill and Génome Québec Innovation Centre, Montreal, Quebec, Canada. Two lanes of Illumina HiSeq2500 RAPID PE250 were used to sequence a TruSeq LT shotgun library with an approximately 380 bp fragment size, and three lanes of Illumina HiSeq 2000 PE100 were used to sequence Nextera Mate Pair libraries targeting 3 kbp, 5 kbp, and 10 kbp sizes.

PacBio library preparation and sequencing was performed by the Norwegian Sequencing Centre, University of Oslo, Norway. Three libraries were prepared using the Pacific Biosciences 20 kbp library preparation protocol, with final library size selection of >7 kbp using BluePippin (Sage Science). All samples were sequenced on a Pacific Biosciences RS II instrument using P6-C4 chemistry. Eight SMRT cells used a four hour movie and 37 cells used a six hour movie, for a total of 45 SMRT cells.

#### Assembly and scaffolding

The ALLPATHS-LG (release 52488) [42] program was used to assemble the three mate-pair libraries and the overlapping paired-end library into an initial genome assembly. Default parameters were used during assembly except: HAPLOIDIFY was set to True, GENOME_SIZE was set to 3 Gbp, and the CLOSE_UNIPATH_GAPS option was set to False. This latter parameter change resulted in ALLPATHS-LG skipping the CloseUnipathGaps step, which can stall for particular data sets (excluding this step does not normally result in a drop in assembly quality). PBJelly (version 15.8.24) [43] was then used to fill gaps and join scaffolds in the initial assembly using PacBio sequences. Default settings were used for this step. Finally, scaffolds longer than 1,000 bp were further assembled using the SSPACE-LongRead program (version 1.1; default settings) [44] to generate the final scaffold set.

The final scaffolds were ordered into chromosomes based on the genetic map created above, an updated male and female genetic map from [15], and synteny with the rainbow trout reference genome assembly (NCBI accession: GCA_002163495.1), similar to the methodology in [27]. All of the perl or python scripts used for this step are included in S1 File. Synteny was only used to place scaffolds if there was concordance with one of the genetic maps.

The genetic marker sequences, from each of the genetic maps, were first aligned to the Arctic charr scaffolds and the rainbow trout genome assembly using BWA mem with default settings and Megablast in BLAST version 2.2.31+ [45,46] (-outfmt 6, -max_hsps 2, -max_target_seqs 4, and -evalue 0.01). The alignments were filtered based on the number of times the sequences aligned to the genome assembly (only one best alignment was retained). The BLAST alignments were filtered using a minimum percent identity (96% for the current genetic map and 94% for the genetic map from a different study), alignment length (143 bp for current map and 63 bp for other maps), and difference in bit score between the best and second best alignment for a marker (10 bits for the current map and 5 bits for the other maps). Different filtering parameters were used for the different genetic maps because the genetic marker sequences were of different lengths (144 bp for current map and a variable length for the other maps 38–85 bp with an average of 71 bp). The lower thresholds were used for the shorter sequences so that they would not be immediately filtered by the more stringent parameters used in filtering the longer sequences.

The Arctic charr scaffolds were aligned to the rainbow trout genome assembly using nucmer version 3.1 in Mummer [47]. These alignments were filtered and required a minimum alignment length of 250 bp and a minimum percent identity of 92%. They were also filtered based on linearity (the scaffold alignment positions needed to increase or decrease accordingly with an increase or decrease of the rainbow trout chromosome positions) using a custom script (Clean_Combined_Genetic_Map_Info_version_1.0.py, S1 File). The linear alignments were filtered based on: maximum distance allowed between chromosomal positions of two alignments (cmax = 0.5% total length of chromosome), maximum distance allowed between scaffold positions of two alignments (smax = 5% total length of scaffold), a minimum total length of linear alignments relative to scaffold length (minl = 10% of the total length of a scaffold), and the minimum total length of linear alignments (minal = 3,000 bp). The same options were used to filter alignments between genome assemblies based on linearity below.

Information from the genetic marker alignments and the synteny information from the Arctic charr scaffold alignments to the rainbow trout genome assembly were next combined for each genetic map. This combination was then used to manually order the Arctic charr scaffolds (see the S1 File for more details). Potential chimeric scaffolds were broken manually. A final quality control was performed, where all genetic markers were aligned to the Arctic charr scaffolds with minor filtering (minimum percent identity 94, minimum alignment length 140) to verify the order and orientation of each scaffold and to add scaffolds without synteny (but with sufficient genetic map information).

### Genome assembly analyses

#### Completeness

A benchmarking universal single copy orthologs (BUSCO) version 3.0.2 [48] analysis was performed to quantify the completeness of the genome assembly before scaffolds were placed onto chromosomes. The actinopterygii_odb9 lineage data set, which was used for this analysis, contains 4,584 BUSCOs from twenty species. The following parameters were used: -m genome, -c 10, -sp zebrafish.

#### Homeologous block identification

SyMAP v4.2 [49] was used to identify homeologous (duplicated) regions/blocks within a repeat-masked version of the Arctic charr genome assembly using the following parameters: merge_blocks = 1, nucmer_only = 1, mindots = 10. The identified blocks were filtered if they had fewer than 100 hits. The orientations of these blocks relative to one another were identified by first filtering the anchors identified with SyMap. The anchors were filtered based on linearity (combined linear alignments needed to be at least 2000 bp long, similar to the method used in *Assembly and scaffolding*) using a custom script (S1 File). After filtering, the number of individual anchors in forward and reverse orientation were counted, and the orientation with the most counts was used as the orientation for a block. The percent identity was also calculated for 1 Mbp windows between homeologous blocks after filtering using custom scripts (S1 File).

#### Repetitive elements

An Arctic charr repeat library was generated following a methodology similar to that found in [26], and the same as in [27]. Briefly, Salmoniformes repeat sequences were obtained from existing sources [26,50] as well as from a *de novo* library generated from an initial Arctic charr assembly using RepeatModeler v1.0.8 [51]. All preliminary library sequences subsequently underwent a process of validation, redundancy removal, non-transposable element (TE) host gene removal, and classification.

The preliminary repetitive sequences were aligned to the Arctic charr assembly using BLAST in order to validate their repetitiveness within the Arctic charr genome (BLASTN word_size = 7). Sequences with fragments occurring in at least three locations across the genome were retained; all others were excluded (for full details, please see [27]). Following repetitiveness validation, an all-by-all BLASTN approach was used to remove redundant sequences wherever more than 80% of a shorter sequence was covered by high-scoring segment pairs from another, longer sequence.

The repetitive sequences that remained in the library were then filtered to remove non-TE host genes and then annotated, using the same methodology as in [27]. Non-TE host genes were identified as those which had a higher-scoring BLASTX hit to a non-TE Swiss-Prot UniprotKB database sequence than to a sequence from the REPET-formatted RepBase v20.05 collection of reference TE proteins.

Repeat classification was guided by the taxonomic system proposed by Wicker et al. [52]. Sequences were first classified to the superfamily level if they had a BLASTN or BLASTX alignment to either the REPET-formatted RepBase v20.05 nucleotide or protein databases (BLASTN: ≥ 80% similarity and ≥ 80% sequence coverage; BLASTX: E-value ≤ 1e-10). The PASTE Classifier tool [53,54] was used to identify potentially chimeric sequences, rDNA sequences (which were removed as non-TE host genes), and miniature inverted-repeat transposable elements. All sequences were examined by dotplot and those which were predominantly composed of satellite or simple repeat motifs were labelled as such.

RepeatMasker version 4.0.7 [55] (options: -gff, -x, and -excln), RMBlast version 2.2.28+, and Tandem Repeats Finder 4.09 [56] were used to mask the Arctic charr genome assembly with the newly created repetitive sequence library. Genomic repetitive element composition was calculated using the RepeatMasker output file (.out file). Following repeat-derived sequence identification using RepeatMasker, the landscape of repeat content variation across the genome was determined. For 1 Mbp windows, the proportion of DNA derived from repeated sequence was calculated as the percent of X’s (output from repeat masking the genome assembly) in those windows using a custom script (S1 File). This information was used in combination with Circos [57] to visualize the repetitive DNA across the genome assembly.

#### Genomic comparisons

The genome assemblies of Atlantic salmon (NCBI accession: GCF_000233375.1), coho salmon (NCBI accession: GCF_002021735.1), and northern pike (NCBI accession: GCF_000721915.3) were compared to the Arctic charr genome assembly (a draft version). The other genome assemblies were first aligned to the Arctic charr genome assembly with Megablast using the following parameters: -evalue 0.0001, -max_target_seqs 3, -max_hsps 20000, -outfmt 6, -word_size 40, and -perc_identity 70. The alignments were then filtered based on linearity using custom python scripts (Compare_Genome_2_Other_Genome_blastfmt6_ver1.0.py, S1 File) (smax 0.01, cmax 0.01, minl 0.01, minal 50000 for Atlantic and coho salmon, and minal of 15000 for northern pike—see *Assembly and scaffolding* section for more details on these parameters). Figures were generated using ggplot2 in R. The chromosomal alignments were compared to the results from [14] to characterize chromosomal arms of the Arctic charr relative to other species. As in [14], each northern pike chromosome was treated as two since salmonids are expected to have multiple homologous chromosomes per pike chromosome due to genome duplication.

#### RNA-seq and gene annotation

Please see the *Samples and library preparation* section for sample information and a list of sampled tissues. RNA was extracted from all tissues using TRIZOL in combination with a RNeasy kit (QIAGEN). RNA samples were then sent to BGI at UC Davis, where RNA-seq libraries were generated and sequenced on an Illumina HiSeq 2000 instrument (PE 100). The raw sequences were then deposited in the NCBI sequence read archive (SRS2043860—SRS2043871). These libraries were submitted to supplement existing RNA-seq libraries to be used in a standardized NCBI Eukaryotic Genome Annotation Pipeline [58].

#### Orthology analysis

In order to identify orthologous genes between species, sets of homologous chromosomes were first identified between species (similar to [59,60]). Protein alignments that passed filtering were used to identify potential orthologous genes on the homologous chromosomes if a putative protein ortholog unambiguously aligned between the two regions a single time. The corresponding genes were called orthologs. Duplicated genes, arising from the ancestral salmonid genome duplication (homeologs), were identified using a similar approach. The following paragraphs detail this procedure.

In addition to the genome assemblies used in the *Assembly and scaffolding* and *Genomic comparisons* sections (Atlantic salmon, rainbow trout, coho salmon, and northern pike), two additional genome assemblies were downloaded from the NCBI: Arctic charr (version annotated by the NCBI and used only for this section, NCBI accession: GCF_002910315.2), and Chinook salmon (GCF_002872995.1). Associated gene annotation files (gff) and protein sequence fasta files were also downloaded for each genome assembly. The genome assembly fasta files were indexed with the faidx command in SAMtools [61], and the Arctic charr proteins were processed with Blast2GO (version 5 Basic) [62] to identify gene ontology (GO) terms. Blast2GO utilized the UniProtKB (Swiss-Prot) database (downloaded on March 28, 2018). Within Blast2GO, all UniProtKB proteins were aligned to the Arctic charr protein set using BLASTP-fast (maximum hits 10, with all other parameters default). Blast2GO’s default mapping and annotation steps were performed after the alignment step and an .annot file (S2 File) was output.

Scaffolds that were not placed onto chromosomes were filtered from the Arctic charr genome assembly sequences using the faidx command in SAMtools (in the bash terminal, the following command was used: for i in {38..76}; do samtools faidx GCF_002910315.2_ASM291031v2_genomic.fna "NC_0368"$i".1" > "NC_0368"$i".1.fasta"; done). The chromosomes were then repeat masked with RepeatMasker (-gff, -excln).

A repeat masked Arctic charr genome assembly BLAST database was generated (makeblastdb) and all genomes (including that of Arctic charr) were aligned to this database using Megablast with the following shared parameters: -outfmt 6, -max_target_seqs 3, and -max_hsps 20000. Parameters for evalue, word_size, and perc_identity varied between genome assemblies as follows: -evalue 0.0001 -word_size 40, -perc_identity 90 (coho salmon, Chinook salmon, rainbow trout), -evalue 0.001, -word_size 35, and -perc_identity 75 (northern pike), -word_size 42, and -perc_identity 94 (Atlantic salmon), and -evalue 0.001, -word_size 35, -percent_identity 80 (Arctic charr). Other values were evaluated, however, those outlined here were used as they produced long orthologous alignments and produced fewer apparently spurious alignments. These alignments were then filtered based on linearity using a python script (S1 File) with -minl 0.01 and -minal 30000 (except for the Arctic charr and northern pike alignments, which had a -minal of 15000) (see *Assembly and scaffolding* section for more details on parameters). An additional filtering step removed overlapping alignments between the genome assemblies using a custom script (S1 File) except for the northern pike and Arctic charr genome assemblies. Alignments to one of the Atlantic salmon chromosomes were removed manually after inspection (between NC_027319.1 and NC_036862.1 near the beginning of the chromosomes) as these alignments created an artificially large orthologous chromosome section. The resulting aligned chromosome regions represented blocks of orthologous chromosome sequence between Arctic charr and other species.

An Arctic charr protein database was generated (makeblastdb) and proteins from each species were aligned to the database using BLASTP and the following parameters: -max_target_seqs 3, -max_hsps 4, -evalue 0.001. These values were used to reduce the number of off-target alignments. BLASTP alignments were further filtered using a python script (S1 File) based on a minimum alignment length of 80% of the total length of each protein, and a minimum average percent identity of 80%. Other values were evaluated, but reductions in the minimum average percent identity and percent of length only slightly increased the number of orthologs.

Following the identification of filtered BLASTP-paired proteins between species, a python script (S1 File) was used to establish which of these pairs represented true orthologs. First, NCBI GFF files (gene annotation files) were used to identify the position of the genes corresponding to each protein within the genome assemblies of the corresponding species. If the genes corresponding to each protein in a pair were located in previously identified orthologous chromosome regions, and if there was only one such pair for each protein, the proteins/genes were labelled as orthologous. The pairwise orthologs were then used to create a table of orthologous genes for all species (S1 Table), which also includes gene duplication information.

#### Gene expression (RNA-seq)

In addition to finding orthologous genes between species, a gene expression analysis was performed to identify genes that had unique tissue expression profiles between species in an effort to identify genes that have diverged, in gene expression patterns, since the most common ancestor of the species. Such genes have a greater likelihood of influencing divergent phenotypes (e.g. semelparity vs iteroparity) between lineages.

For Arctic charr, Chinook salmon, coho salmon, Atlantic salmon, northern pike, and rainbow trout, paired-end RNA-seq sequences (see Table 2 for NCBI accessions) were imported into CLC Genomics Workbench 9.5.4 [63]. The following options were used for the import: minimum distance 1, maximum distance 900, and remove failed reads. Next, the reads were mapped to their corresponding genome assemblies with the following options: map to gene and intergenic regions, mismatch cost 2, insertion cost 3, deletion cost 3, length fraction 0.8, similarity fraction 0.92, maximum number of hits 1, expression value reads per kilobase of gene per million mapped reads (RPKM), calculate RPKM for genes without transcripts, and use expectation-maximization estimation (in the CLC software, fragments per kilobase of gene per million mapped reads, or FPKM, is reported as RPKM, but the default output is for FPKM).

**Table 2:** NCBI accessions for RNA-seq analysis.

Species	Tissue	NCBI (SRA) Accession
**S. alpinus, O. tshawytscha, O. kisutch, S. salar, E. lucius, O. mykiss**	Brain	SRX2635054, SRX3379484, SRX2632051, SRX608607, SRX514235, SRX2894156
	Eye	SRX2635059, SRX3379482, SRX2632050, SRX608616, SRX514236, NA
	Gill	SRX2635050, SRX3379485, SRX2632049, SRX608399, SRX514237, SRX2894158
	Gonad	SRX2635049, SRX3379473, SRX2632041, SRX608620, SRX514271, SRX2894150
	Gut	SRX2635056, SRX3379477, SRX2632048, SRX608567, SRX514238, SRX2894160
	Head Kidney	SRX2635052, SRX3379472, SRX2632047, SRX608569, SRX514240, SRX2894157
	Heart	SRX2635058, SRX3379476, SRX2632046, SRX608571, SRX514258, NA
	Hind Kidney	SRX2635053, NA, SRX2632045, SRX608574, SRX514263, SRX2894159
	Liver	SRX2635048, SRX3379480, SRX2632044, SRX608575, SRX514266, SRX2894162
	Muscle	SRX2635055, SRX3379475, SRX2632043, SRX608579, SRX514267, SRX2894153
	Spleen	SRX2635057, SRX3379469, SRX2632038, SRX608599, SRX514270, SRX2894163
	Stomach	SRX2635051, SRX3379470, SRX2632037, NA, SRX514269, SRX2894151

Accession numbers are ordered by species from the species column

Gene expression values were assembled into a table for each species (S2 Table—rows correspond to those in S1 Table) using custom python scripts (S1 File). These tables were imported into R, where a pseudo-value of 0.01 was added to the expression values and the sum was log10 normalized, as in [64]. Similar to [64], correlations between tissues (within and among species) were found using the ‘cor’ function (for the set of 5304 overlapping orthologs of all species and homeologs), which calculates the Pearson correlation coefficient by default (see S1 Fig for a graphical representation). The heatmap.plus R package [65] and the heatmap.2 function in the ‘gplots’ R package [66] were used to visualize and group tissues by correlation coefficients (for complete R code, see S1 File).

To identify genes that have unique expression patterns in Arctic charr when compared to the other salmonids in this study, correlation values were calculated between Arctic charr and the other species for each identified ortholog (a subset with known orthologs for all salmonids) using the normalized expression values (as above) with the ‘%>%’ pipe function in the magrittr package [67] in R, as well as the ‘rowwise’, ‘do‘ and ‘cor’ functions (see S1 File for more details and S1 Fig for a visual representation) (similar to [26]). Together, these functions produced a new column with the correlation values between the different tissues of the Arctic charr ortholog and the other species’ ortholog (a different column for each species comparison).

A subset of genes was identified that had correlation coefficients equal to or below the absolute value of 0.5 between Arctic charr and each of the other salmonids in the study (rainbow trout, Atlantic, Chinook, and coho salmon). A value of 0.5 was chosen based on the separation of correlation coefficients using a kmeans clustering method in R with a cluster value set to two. These genes are expected to have a higher likelihood of influencing traits specific to Arctic charr since they have expression patterns that are different from the other salmonid species.

A set of Arctic charr genes that exhibited low correlation coefficients between homeolog pairs was also identified. These genes had correlation coefficient values less than or equal to the absolute of 0.5—based on another kmeans analysis. The genes in this set represent homeologs whose expression patterns have diverged since the genome duplication, and represent possible examples of neofunctionalization or subfunctionalization.

Following identification, both the low-correlation ortholog gene set and the low-correlation homeolog gene set were examined for the enrichment of particular GO terms using a Fisher’s Exact Test in Blast2GO (default settings). As the GO annotation was based on proteins and the gene expression data was based on genes, it was necessary to convert the gene names to protein names using custom scripts (S1 File). It was also necessary to remove redundant protein isoforms, as well as one gene from each homeologous pair (for the second subset) as either case would artificially create significant enrichment categories. This removal was done with custom scripts (S1 File).

#### Nucleotide variation between two commercial strains

Two Tree River (Tree River: TR, Nauyuk Lake: NL), two hybrid individuals (between a TR male and NL female), and four crosses (of various mating strategies: (TRm x (TRm x NLf)f)m x (TRm xNLf)f, NLm x ((TRm x NLf)m x TRf)f, (TRm x NLf)m x NLf, TRm x ((TRm x NLf)m x TRf)f) of Arctic charr were sampled to find nucleotide variants between the Tree River and Nauyuk Lake strains. These fish were obtained from and reared at Icy Waters Limited (Whitehorse, Canada). The DNA extraction followed the same phenol extraction protocol that was performed to obtain DNA for genome sequencing and assembly (see the *Samples and library preparation s*ection). Illumina library preparation (TruSeq LT shotgun 425 bp fragment size) and sequencing was performed by the McGill and Génome Québec Innovation Centre, Montreal, Quebec, Canada. Each library was sequenced on one lane of Illumina HiSeq2500. All animals were reared and sampled in compliance with the Simon Fraser University animal care protocol #1155MB-08.

The Burrows-Wheeler Aligner (bwa aln [68]) was used to align the paired-end reads (without any filtering or trimming), from the eight Arctic charr, to the Arctic charr scaffolds. These scaffolds were from an earlier version of the genome assembly (before scaffolds were placed into chromosomes). Mpileup in SAMtools was used in conjunction with BCFtools (call) to generate SNPs from each of the alignments produced by BWA. SNPs were filtered based on the following criteria: filter = ‘.’, quality score for alternate assertion ≥ 20, RMS mapping quality ≥ 30, genotype quality ≥ 20, 1 ≤ depth ≤ 100.

## Results and discussion

### Genetic map

#### Data processing and genetic map construction

From four ddRAD sequencing libraries, ~401 million filtered reads (~1.2 million per individual) were retained from ~598 million initial reads (~67%) after filtering with Stacks. Following additional filtering and genotype calling with Stacks, 38,837 SNPs were retained. During linkage group construction, 12,645 SNPs were retained at 8,574 loci or ‘stacks’ (S3 File). The SNPs were separated into 39 linkage groups, with a length of 2,724 cM after ordering the markers. These markers were aligned to the final genome assembly sequence to visualize how the present genetic map was used in the assembly, along with the male and female updated genetic map from [15], which were also used in the assembly (S2 Fig).

There are three primary differences between linkage groups in the previous genetic map and the current genetic map: 1) linkage group AC04 from the previous map was split into three linkage groups in the new genetic map, 2) linkage group AC29, from the previous genetic map, was fused with one of the split AC04 linkage groups, and 3) linkage group AC06, from the previous genetic map, was split into two linkage groups. The differences between genetic maps are reflected in the nomenclature of the linkage groups in Fig 1.

**Fig 1:** Circos plot of Arctic charr genome assembly. A) Is comprised of bar charts for each chromosome with the fraction of repetitive DNA found in million bp windows with a scale from 0 to 1 (bars with scores greater than 0.65 are shown in orange). B) Displays bar charts of percent identity between homeologous regions defined by SyMap v4.2. The percent identity was found by weighting the percent identity by alignment lengths. Each bar represents a million bp window, and the y-axis starts at 75 percent and ends at 100 percent identity. Windows with score greater than 90 percent were highlighted orange. C) Ideograms of each of the Arctic charr chromosomes. The internal ribbons link homeologous (or duplicated) regions of the genome.

AC04 has previously been detected as a single linkage group or as two linkage groups depending on mapping parents [15,69]. These discrepancies presumably arise from centric fusions and fissions involving two acrocentric arms. The AC04p chromosome is thought to be the Arctic charr sex chromosome (allosome) [15]. From the association analysis, using the genders from the current mapping families, three significant peaks were found on AC04q.1.29, AC04q.2, and AC04p (S3 Fig).

It seems unlikely that these associations are real and based on the previous genetic map, it seems plausible that AC04q.1.29, AC04q.2, and AC04p may have been erroneously broken (i.e. there is linkage between AC04q.1.29, AC04q.2, and AC04p, and the association on AC04q.2 and AC04p is from markers in linkage disequilibrium to the sex determining region on AC04q.1.29). Further support for AC04p and AC04q.2 belonging to a single linkage group can be found below, as well as conflicting evidence regarding the inclusion of AC04q.1.29 in a linkage group combining all three linkage groups. Plans for future Arctic charr genome assembly updates are underway to resolve these issues and to increase the accuracy of the genome assembly by utilizing sequence polishers.

### Genome assembly

#### Data processing and genome assembly

ALLPATHS-LG estimated a genome size of ~2.4 billion nucleotides for the Arctic charr. From this estimate, the mate-pair libraries each had a genome coverage of between 13-15x (3 kbp– 13.49x, 5 kbp– 14.46x, 10 kbp– 14.73x). The paired-end library had a coverage of around 79x, and the PacBio genome coverage was roughly 26x (average length = 4760.3 bp, N50 = 7629 bp, range = 35 bp—70170 bp). Together the libraries had an estimated coverage of 147.56x. The pre-processed DNA sequences can be found in the NCBI sequence read archive (SRP101753).

After ALLPATHS-LG assembly, there were 29,290 scaffolds with an N50 of around 888 kbp (range: 1,000 bp—10,231,177 bp). PBJelly reduced the number of scaffolds to 24,044 and increased the scaffold N50 to around 914 kbp (range: 887 bp—8,893,364). After SSPACE scaffolding, there were 16,264 scaffolds with roughly 2.2 billion nucleotides (scaffold N50: ~1,168 kbp). Using synteny with the rainbow trout genome assembly in concordance with the genetic maps, 1,486 of these scaffolds were ordered into 39 chromosomes. The 1,486 scaffolds represent ~1.5 billion nucleotides or ~70% of the genome. The final assembly had a scaffold N50 of 1.02 Mbp and the contig N50 was 55.6 kbp (GenBank accession: GCA_002910315.2).

#### Completeness

The BUSCO analysis identified 4,086 complete (89.2%), 129 fragmented (2.8%), and 369 missing (8.0%) BUSCO reference genes out of 4,584. These results were similar to those from the Chinook salmon genome assembly [27], in which researchers found 90.3% complete genes of the same set of BUSCOs used in this study (2.1% fragmented and 7.6% missing). This suggests that most of the genome is present in our assembly.

#### Homeologous block identification

SyMAP identified 168 homeologous blocks originally, but only 78 blocks were retained after filtering those with fewer than 100 anchors. These blocks are shown on a Circos plot in Fig 1. As seen in other salmonids [16,26,70], these regions often have high similarity with their homeologous chromosome counterpart (Fig 1). On average, these homeologous regions had alignments with ~88% similarity (for regions that aligned). A spike in percent similarity was often observed near the ends of chromosomes that likely reflects the high level of recombination that occurs between these homeologous chromosome regions [16]. This pattern follows that seen in Atlantic salmon [26], rainbow trout [70], and Chinook salmon [27].

#### Repetitive elements

RepeatMasker identified 56.38% of the genome (on chromosomes) as being derived from repetitive elements (S3 Table). Class I and Class II TEs make up 18.48% and 21.82% of the Arctic charr genome respectively (S3 Table). Most of the remaining repetitive elements are unclassified (S3 Table). In Mbp windows, across the genome assembly, the average percent of repetitive elements was reflective of the overall percent of repetitive elements (53.76%; with a minimum of 7.48% and a maximum of 75.35%, Fig 1). Again, this pattern follows those seen in other salmonid genome assemblies [26,27].

Several regions of the genome have high levels of repetitive elements (Fig 1). These regions are associated with centromere positions in Atlantic and Chinook salmon [26,27], and thus could represent centromeres here. Given that the position of centromeres may change over time, these regions may not reflect current centromere positions [71]. These positions will need to be confirmed with other approaches such as centromere mapping [17,72,73].

#### Genomic comparisons

A comparison of whole genome alignments in Arctic charr and other species suggests that there are relatively few chromosomal rearrangements between Arctic charr and other species from the Salmonidae family compared to the number found between the Arctic charr and the northern pike (Fig 2). As expected, there are two Arctic charr chromosomes for every northern pike chromosome (Fig 2, Table 3, S4 Fig). A considerable difference between the Arctic charr chromosomes and those from other salmonids in this study, is that the majority of the charr’s homologous chromosomes show one-to-one relationships with the northern pike chromosomes (Table 3).

**Fig 2:** Comparison of genome assemblies from selected species to the Arctic charr genome assembly. The lighter colors represent alignments that are in forward orientation, while the darker colors represent reverse orientations. For the Arctic charr chromosomes, all numbers indicate corresponding chromosome names without the prefix of AC (and 0 for those below 10). For all other species, the chromosome numbers represent NCBI designations without letter prefixes.

**Table 3:** Homologous chromosome arm comparison between species.

E. lucius (pike)	S. alpinus (charr)	O. kisutch (coho)	S. salar (Atlantic)
1.1	**AC22**	15b	20b
1.2	**AC04p**	18a	9c
2.1	AC15b	3b	**26**
2.2	**AC10**	8b	11a
3.1	**AC32**	**30**	14a
3.2	**AC19**	**27**	3a
4.1	AC08a	15a	9b^c^
4.2	**AC06.2**	19b	5a
5.1	AC18a	20a	19b
5.2	AC08b	**25**	**28**
6.1	AC18b	11a	1b
6.2	**AC25**	4b	18a
7.1	AC20b	6a	13b
7.2	**AC23**	**28**	4b
8.1	AC13b	10a	**23**
8.2	**AC16**	13a	10a
9.1	**AC21**	20b	2b
9.2	AC01a	1b	12a
10.1	**AC31**	17a	**27**
10.2	**AC30**	14b	14b
11.1	AC20a	10b	6a
11.2	AC20d	6b	3b
12.1	**AC17**	**24**	13a
12.2	**AC07**	17b	15b
13.1	AC15a	3a	**24**
13.2	**AC33**	8a	20a
14.1	AC04q.1.29a	**23**	1c
14.2	(AC20c, AC28a)^a^	**29**	11b
15.1	**AC04q.2**	14a	9a
15.2	**AC09**	7b	1a
16.1	**AC36**	**26**	**21**
16.2	**AC02**	2b	**25**
17.1	AC01b	1a	12b
17.2	**AC11**	5b	**22**
18.1	AC28b	12a	15a
18.2	AC14a	**21**	6b
19.1	AC04q.1.29b	**22**	10b
19.2	AC26b	4a	16a
20.1	AC06.1a	13b	5b
20.2	**AC35**	2a	2a
21.1	AC27a	11b	**29**
21.2	AC14b	18b	19a
22.1	AC27b	5a^b^	17a
22.2	**AC12**	16b^b^	16b
23.1	AC03a	9a	7b
23.2	**AC24**	19a^c^	17b
24.1	AC03b	9b	7a
24.2	**AC37**	16a	18b
25.1	AC13c	12b	4a
25.2	**AC34**	7a	**8**

A comparison of Arctic charr homologous chromosome arms based on chromosome nomenclature from [14]. For each northern pike chromosome there are two chromosomes in the Salmonidae family due to an early salmonid-specific genome duplication (e.g. 1.1 and 1.2 refer to the same northern pike chromosome).

^a^Expected to align to Arctic charr chromosome AC05, but aligned to AC20c and AC28a.

^b^Appears to be a transposition error based on the current alignments.

^c^9b and 19a did not align with the parameters that were used, and are consequently missing in the current analysis.

Chromosomes that only match one northern pike chromosome are in bold text.

Twenty-five out of 39 Arctic charr chromosomes have a single homologous pike chromosome, compared to the 10 (out 29 for Atlantic and of 30 for coho salmon respectively) found between the other salmonids and northern pike. Similarly, the brook charr (*Salvelinus fontinalis*), a congener of Arctic charr, has 33 (out of 42) single homologous linkage groups when compared to pike [14]. The remaining chromosomes appear to have Robertsonian fusions between ancient acrocentric chromosomes [20]. At least two homologous associations between different Northern Pike chromosomes and a single Arctic charr chromosome would be expected if the Arctic charr chromosome is metacentric in configuration.

These results are consistent with previous cytogenetic analyses of Arctic and brook charr genomes, which both have “A” type karyotypes [20]. The difference between the “A” type karyotype and the “B” type karyotype has been suggested to be related to different rates of recombination (with fewer chromosomes or chromosome arms, there might be fewer recombinations per genome in the “B” type karyotypes), which may impact the rate of local adaptation because adaptive haplotypes have a greater chance to form [20].

The putative sex chromosome (AC04, AC04q.1.29 in the current analysis and AC04p found in a previous study [15]) appears to have been split into three linkage groups in the current study (see above). From the genomic alignments (Fig 2), AC04p and AC04q.2 both align to the Atlantic salmon chromosome 9 (ssa09), further supporting the argument that the two belong to a single linkage group or chromosome. In all other cases, however, AC04q.1.29, AC04p, and AC04q.2 aligned to different chromosomes of the species analyzed. This would suggest that either they belong on different chromosomes, or that there was a lineage-specific chromosomal fusion of these chromosomes.

#### RNA-seq and gene annotation

All RNA-seq data were submitted to the sequence read archive (SRS2043860—SRS2043871). The total number of paired-end reads was ~1.084 billion and averaged ~90 million per tissue (min: 74,929,414 in spleen, max: 106,646,706 in head kidney). For the Arctic charr genome assembly, the NCBI Eukaryotic Genome Annotation Pipeline identified a total of 46,775 genes and pseudogenes, of which 36,435 were protein coding, 5,908 were non-coding, seven were transcribed pseudogenes, and 4,329 were non-transcribed pseudogenes. This annotation approach utilized RNA-seq data from the current and other studies (almost 6 billion reads were used in this annotation, with 77% aligning to the Arctic charr genome assembly) [74]. Of the salmonid genome assemblies that have been annotated with the same pipeline, Arctic charr has the second smallest number of genes/pseudogenes, with only coho salmon possessing fewer; Atlantic salmon have 57,783, rainbow trout have 55,630, Chinook salmon have 53,685, and coho salmon have 46,096 [75–78]. In order to facilitate future comparisons, RefSeq gene annotations and accessions were used in the *Orthology analysis* and *Gene expression (RNA-seq)* sections (below).

#### Orthology analysis

Homologous (or orthologous) chromosome pairs were identified between all but three Arctic charr chromosomes and chromosomes from northern pike, Atlantic salmon, rainbow trout, coho salmon, and Chinook salmon (S5 Fig). No ortholog to Arctic charr chromosome NC_036864.1 (AC24) was identified in coho salmon, and no orthologs to Arctic charr chromosomes NC_036860.1 (AC20) and NC_036874.1 (AC35) were identified in Chinook salmon. The missing orthologs were attributed to high sequence similarity between homeologous chromosomes and our inability to unambiguously assign one of them to a particular orthologous chromosome. To show the extent of the identified orthologous regions, an example of the orthologous chromosome alignments can be seen between the Arctic charr and the rainbow trout genome assemblies (Fig 3).

**Fig 3:** Example of homologous chromosomes and orthologs between species. Linear alignments between the rainbow trout and Arctic charr genome assembliess are shown in the bottom graph. The rainbow trout chromosomes correspond to the NCBI RefSeq accession from the lowest number to highest. Identified orthologous genes are plotted with their relative positions on the rainbow trout and Arctic charr chromosomes on the top graph. Genes without a known ortholog are plotted in gray.

The ability to identify distinct orthologous sequence pairs between salmonid species using a similarity-based approach, even in the presence of potentially confounding homeologous regions, implies that in the majority of cases, diploidization likely occurred before speciation. Were this not the case, both homeologous chromosomes in species A would have approximately the same similarity to a chromosome in species B, and no distinct ortholog pair would have been uniquely identifiable. This observation only applies to the specific orthologous regions we identified herein; it does not, for example, preclude the existence of other regions which underwent diploidization following lineage diversification (see [79] for a discussion on lineage-specific differentiation).

Once orthologous regions were defined, corresponding protein alignments were used to identify orthologous genes between the species (Fig 3). An example is shown to illustrate that the majority of identified orthologous chromosomes share extensive synteny (Fig 3). The maximum number of orthologs identified between Arctic charr and another species was 19,646 for rainbow trout, and the lowest was 15,805 for northern pike (Table 4). For the preponderance of genes with identified orthologs, most of the orthologs were identified for all salmonid species (Table 4, Fig 4). The NCBI annotated 46,775 (36,435 protein-coding) genes in the Arctic charr genome assembly, with 27,172 protein-coding genes placed on chromosomes. Of the possible 27,172 orthologs that could be identified using the methodology presented here, at the high end ~72% of them were identified in rainbow trout and at the low end ~58% of the orthologs were identified between Arctic charr and northern pike.

**Table 4:** Number of identified orthologs between Arctic charr and other species.

Species	Orthologs
Arctic charr	11,252 (homeologs)
Northern pike	15,805
Chinook salmon	16,709
Coho salmon	17,837
Rainbow trout	19,646
Atlantic salmon	18,252

**Fig 4:** Overlapping orthologs and homeologs between species. A histogram of the number of species with a specific ortholog. If an ortholog was found in all species (including homeologs), it would be in the ‘Homeologs and Orthologs’ column. If an ortholog/homeolog was found in four species, it would be in the 4+ column and all prior columns. The ‘All Orthologs’ column contains only the overlapping orthologs (without regards to overlap with a homeolog) of all the species in this study. Likewise, the ‘All Salmonid Orthologs’ column contains the count of overlapping orthologs (and not homeologs) in only the salmonid species (Arctic charr, rainbow trout, coho salmon, Chinook salmon, and Atlantic salmon).

Only 11,252 homeologous genes were found between the Arctic charr homeologous chromosomes (Table 4). Many homeologs can be expected to have been lost during diploidization, and this may partially explain the lower observed number of homeologs. In the Atlantic salmon genome assembly, 56% of the analyzed singleton genes had pseudogenized homeolog gene fragments in syntenic homeologous genome locations instead of whole genes [26]. Such homeolog fragments would likely not be identified as a homeolog in the current analysis. The current set of homeologous genes represents around 41% of the 27,172 protein-coding genes on chromosomes. This is similar to the 48% of duplicated genes that were found in the rainbow trout genome assembly [70].

#### Gene expression (RNA-seq)

Overall, ~72% of RNA-seq reads aligned to their respective genome assemblies (74% for Arctic charr) (Table 5). These alignments were used to calculate the fragments per kilobase of gene per million mapped reads (FPKM) for various tissues (Table 2). Caution should be taken when evaluating these results; the FPKM values were generated from only a single individual at a single time-point for each species (S2 Table—expression data in rows correspond to the genes in S1 Table). These data are reported and evaluated on the basis of hypothesis generation only.

**Table 5:** RNA-seq statistics.

Species	Average Total Reads	Average Percent Mapped
Arctic charr	90,405,878	74
northern pike	59,880,079	80
coho salmon	205,322,058	72
rainbow trout	89,299,071	65
Atlantic salmon	61,971,752	74
Chinook salmon	256,708,646	69

Expression values were first analyzed by comparing tissues between species using the correlation of all overlapping orthologs in those tissues, and then by identifying genes that had low tissue correlation between Arctic charr and either the other salmonid species or homeologous genes (S1 Fig). The distributions of correlation coefficients (based on gene expression patterns of various tissues between orthologs—Table 2), between Arctic charr and the other species/homeologs, all suggest that the majority of orthologs and homeologs have very similar gene expression patterns (Fig 5). Similar gene expression patterns between orthologs are expected, which lends greater credence to the ortholog assignments. A greater percentage of orthologs between Arctic charr and other salmonid species have highly similar expression patterns than do homeologous gene pairs or orthologs between Arctic charr and northern pike (Fig 5). The only exception is the rainbow trout, which had two missing tissues (Table 2) that may account for the lower correlation coefficients.

**Fig 5:** Histograms of correlation coefficients found between Arctic charr orthologs and other species. Each histogram also has a pie diagram to illustrate the frequency of a range of correlation values. Each histogram is labeled for the species that was compared to the Arctic charr orthologs (SalpH—11,035 homeologous genes, Eluc—15,428 orthologous northern pike genes, Okis—17,490 orthologous coho salmon genes, Otsh—16,320 orthologous Chinook salmon genes, Ssal—17,617 orthologous Atlantic salmon genes, Omyk—19,122 orthologous rainbow trout genes).

The distribution of correlation coefficients, based on gene expression patterns between homeologs, within the Arctic charr genome assembly is similar to the distribution between Arctic charr and northern pike orthologs, although the northern pike still had fewer highly correlated orthologs than the homeologs (Fig 5). The other salmonid species had greater similarity to Arctic charr than did the comparisons with Northern pike. The divergence times between salmonid species, the divergence time between Arctic charr and northern pike, and the timing of the salmonid specific genome duplication may shed light onto why the distributions were different.

Differences in the time that has passed since the founding event (either speciation or whole genome duplication) for a group of homologous genes may explain the differences which occur between the correlation coefficient distributions of Arctic charr homeologs, Arctic charr-salmonid orthologs, and Arctic charr-northern pike orthologs. The time since the most common ancestor of Arctic charr and Northern pike is estimated to be approximately 113–140 MYA [13,80], while the salmonid-specific whole genome duplication is believed to have occurred ~90 MYA [13]. In comparison, the split between the *Salvelinus*, *Oncorhynchus*, and *Salmo* genera occurred roughly 14 MYA [13]. Under this paradigm, orthologs between Arctic charr and northern pike would exhibit the least similar expression profiles because they have had the most time to diverge from each other. Homeologs arising from the whole genome duplication would be expected to possess more highly correlated expression profiles than the northern pike orthologs, and expression profiles between salmonid orthologs would be expected to be the most similar.

At the tissue level, the eye, brain, gonad (either testis or ovary), muscle, and liver grouped well into separate clades based on gene expression correlation coefficients found between each tissue for most of the species evaluated (Fig 6). The gut, stomach, and gill tissues clustered well for most of the salmonids. Most of the homeologous genes, northern pike, and Chinook salmon tissues formed their own separate clades. This would suggest that variance in gene expression among tissues was less within these species than the variance to corresponding tissues in different species. These clades should be interpreted with caution, as they may form from a subset of genes with uncontrolled gene expression, and with species comparisons some genes will be tissue-variable while others will be species-variable [64].

**Fig 6:** Heatmap of correlation coefficients between species and tissues. Pearson correlation coefficients were calculated between different tissues and species combinations based on log transformed gene expression values (5304 common orthologous or homeologous genes). These values were then used to cluster each tissue-species combination. Both dendrograms represent the same information and each leaf depicts one tissue and species combination. The heatmap shows the correlation coefficient between each combination. The groups at the bottom were manually added to help show how the groups were clustered. (Salp—Arctic charr, SalpH—Arctic charr homeologous gene pair, Okis—coho salmon, Otsh—Chinook salmon, Ssal—Atlantic salmon, Eluc—northern pike, Omyk—rainbow trout).

Overall, gene expression was highly correlated between orthologs in the same tissues from different species (Fig 5, S6 Fig), however, the genes with different expression patterns between tissues may be of particular interest since they are more likely to influence differing traits between species. To identify genes that have a greater likelihood of influencing traits unique to Arctic charr, genes were identified that had low gene expression correlation coefficients between all salmonid species in this study and Arctic charr. By comparing all of the salmonid species, environmental influenced differences should be reduced, but not removed. In total, 351 genes were identified that have low correlation coefficients (less than or equal to the absolute value of 0.5) (S4 File). A GO term enrichment analysis was performed to identify any over-represented gene categories (330 proteins were used as they had GO terms—only one isoform was used). There were 10 enriched GO terms (S5 File).

The most significant term from the biological process category was the mitochondrial respiratory chain complex assembly. The most significant cellular component and molecular function category terms were photoreceptor disc membrane and structural constituent of eye lens, respectively. The mitochondrial enriched term is intriguing as increased mitochondria density has been observed in muscle cells of Antarctic fishes [81] and the mitochondrial genome may play a role in thermosensitivity [82,83]. Likewise, the GO terms related to the eye are interesting as the Arctic has a much different light environment than other regions, and Arctic organisms would need to adapt to extended low light conditions [84] and potentially to higher UV exposure [85].

In a similar analysis, 2,887 Arctic charr genes, with low gene expression correlation coefficients between their homeologous gene, were identified (1,375 proteins excluding isoforms and only having one homeolog represented) (S4 File). Homeologous genes with divergent gene expression patterns are likely examples of genes that have neofunctionalized or subfunctionalized (though more likely neofunctionalized [26]), and have escaped diploidization. A GO term enrichment analysis was performed to identify categories of genes that likely escaped diploidization through one of these mechanisms. From this analysis, 109 GO terms were enriched (S5 File).

The most significant biological process category was cell communication, and 753 of the 1,375 (~55%) proteins belonged to this category. Many of the other categories were related to signalling, metabolism, regulation, and ion transport. These results are consistent with Atlantic salmon homeologs, and would suggest dosage plays a significant role in homeolog retention as suggested elsewhere [26,86]. The most significant cellular component GO term was integral component of membrane, with 394 proteins, and the most significant molecular function GO term was the alpha-adrenergic receptor activity, with 6 proteins.

The identified GO categories are likely influenced by environmental variables. For example, if a homeologous gene pair is not expressed under a specific condition/environment, it would not be identified as having a divergent gene expression pattern. The homeologous gene pairs identified here would still likely be examples of neofunctionalization or subfunctionalization (as they have diverged at least in the current conditions), but more homeologs might be added. This could create more enriched GO categories, but would be less likely to remove the current GO categories (the p-value is calculated using a Fisher’s exact test and each additional homeologous pair would likely only slightly change the contingency table).

#### Nucleotide variation between two commercial strains

As an initial assessment of nucleotide variation that can exist between two strains of Arctic charr, resequencing (mean coverage = 21.96 +/- 66.02) was performed for several individuals from various crosses. Nucleotide variants were then identified for each individual (Table 6). Around 4–5 million SNPs were identified from Arctic charr of the Tree River strain and nearly double that number (8–9 million SNPs) were found in hybrid individuals between Tree River and Nauyuk Lake (TR x NL). An intermediate number of SNPs were found between the other more complex crosses between TR and NL. Though a direct comparison between the Tree River and Nauyuk Lake strains was not performed, the relative numbers of SNPs between the Tree River strain and the crosses suggests that the strains vary greatly and reflects the great diversity that exists in Arctic charr [87].

**Table 6:** Number of SNPs identified in commercial stains of Arctic charr.

Genetic Background	Heterozygous SNPs	Total Nucleotide Variants	SNP Frequency / kbp
Tree River	2986470	4355891	2.03
Tree River	3322237	4649645	2.16
TRm x NLf	7222605	8573274	3.99
TRm x NLf	7413500	8715877	4.05
(TRm x (TRm x NLf)f)m x (TRm xNLf)f	5686470	7681273	3.57
NLm x ((TRm x NLf)m x TRf)f	6214612	8497451	3.95
(TRm x NLf)m x NLf	4665517	8227761	3.83
TRm x ((TRm x NLf)m x TRf)f	4688898	5906707	2.75

## Conclusions

The Arctic charr genome assembly represents the first published and publicly available “A” type karyotype genome and opens the possibility of future analyses in the evolution of the salmonids. In this study, we have identified a large number of orthologs between salmonid species and northern pike (a sister taxon) and demonstrated one possible use of this type of data by identifying genes that are more likely to be involved in speciation. The genome assembly sequence will hopefully facilitate further studies on their unique physiology, commercially important traits, and genomic comparisons between different groups of salmonids.

## Supporting information

S1 Fig Methodology of gene expression analyses between species. Two analyses were performed using the orthologous gene expression data and both are illustrated in this figure. A) In this example, there are three species (Arctic charr, Chinook salmon, and coho salmon) and there are three orthologous genes found between all three species with expression data (Genes 1–3). B) The tissue analysis compared tissue gene expression between species and tissues. Each column from A) was compared to each other column to identify the correlation coefficient between them. The resulting correlation coefficient matrix was then used to organize the tissues. C) To identify genes with divergent gene expression patterns, a correlation coefficient was calculated between each species and Arctic charr for each gene based on its expression in the various tissues of the two species. All values are for illustration only.
(PDF)

S2 Fig Comparisons between the current genetic map (genetic map 1) and the previous female (genetic map 2) and male (genetic map 3) genetic maps from an updated version of [15]. On each page, the genetic maps were aligned to a single chromosome. The names for each chromosome were taken from the previous genetic maps.
(PDF)

S3 Fig A manhattan plot of a genome wide association analysis for gender. On the y-axis, the -log10(p-value) is plotted for each of the Arctic charr linkage groups on the x-axis. The blue line represents the Bonferroni corrected alpha level of 0.05 and the red line represents the corrected 0.01 alpha level. The x-axis is labeled by original linkage group name. AC04q.1.29 corresponds to linkage group 4, AC04p corresponds to linkage group 34, and AC04q.2 corresponds to linkage group 35.
(PDF)

S4 Fig A comparison of genome assemblies from selected species to the Arctic charr genome assembly (in a larger format than Fig 2). The darker colors represents alignments that are in reverse orientation, while the lighter colors represent forward orientations.
(PDF)

S5 Fig A comparison of genome assemblies from selected species to the Arctic charr genome (NCBI version), which were used to define orthologous regions of the genome. For each figure, the alignment information is included, and any chromosomes that were lost between the two species are shown with a red arrow. Please see the o*rthology analysis* section to identify which chromosomes correspond to the red arrows.
(PDF)

S6 Fig A heatmap of correlation coefficients between all species and tissues. Only correlations equal to or greater than 0.5 are shown (others are shown as gray). A subset of only salmonid genes are shown on the second page. The number of orthologs used in each analysis is shown at the top. (SalpH—homeologous genes, Eluc—northern pike, Okis—coho salmon, Otsh—Chinook salmon, Ssal—Atlantic salmon, Omyk—rainbow trout).
(PDF)

S1 Table A list of all the genes in the Arctic charr genome assembly and their corresponding orthologs or homeologs for other species. This file is a compressed tab-delimited file.
(GZ) Click here for additional data file.

S2 Table Gene expression values corresponding to the genes from S1 Table. There is one file for each species and a column in each for a different tissue. The files are tab-delimited and are compressed. Each row corresponds to the same row in the S1 Table.
(GZ) Click here for additional data file.

S3 Table Categories and counts of various repeat elements found in the Arctic charr genome. The file is a compressed document file.
(GZ) Click here for additional data file.

S1 File Perl and python scripts used in this study. These files are compressed. Please refer to the readme file for more information regarding any of the scripts and for more information. The readme file also contains R code.
(GZ) Click here for additional data file.

S2 File Arctic charr protein GO annotations. This file is compressed and in Blast2GO format. It has the GO term annotations of all the proteins in the Arctic charr genome assembly (only one isoform was retained in this file).
(GZ) Click here for additional data file.

S3 File Arctic charr genetic map generated from this study. This file is a compressed spreadsheet file.
(GZ) Click here for additional data file.

S4 File The genes that were identified to have low correlation coefficients between Arctic charr and the other salmonids. This file also contains the genes with low correlation coefficients between Arctic charr homeologs. This file is a compressed tab-delimited file.
(GZ) Click here for additional data file.

S5 File Enriched GO categories of genes with low correlation coefficients (0.5). This file is a compressed spreadsheet file.
(GZ) Click here for additional data file.
